# VEGFA-Enriched Exosomes from Tendon-Derived Stem Cells Facilitate Tenocyte Differentiation, Migration, and Transition to a Fibroblastic Phenotype

**DOI:** 10.1155/2022/8537959

**Published:** 2022-09-09

**Authors:** Zhaowen Xue, Zihang Chen, Tingting Wu, Riwang Li, Chao Chen, Junting Liu, Huige Hou, Xiaofei Zheng, Huajun Wang

**Affiliations:** ^1^Department of Bone and Joint Surgery and Sports Medicine Center, The First Affiliated Hospital, Jinan University, Guangzhou 510630, China; ^2^Department of Orthopedics, School of Traditional Chinese Medicine, Southern Medical University, Guangzhou 510515, China; ^3^Department of Orthopedic Trauma and Hand Surgery, The First Affiliated Hospital of Guangxi Medical University, Nanning 530021, China

## Abstract

Tendon-derived stem cells (TDSCs) play a vital role in repair of rotator cuff tear injuries by secreting paracrine proteins that regulate resident cell functions. Secreted exosomes may play a role in tendon injury repair by mediating intercellular communication; however, the detailed mechanisms by which TDSC-derived exosomes affect tenocyte development remain unknown. Here, we examined the effects of exosomes isolated from conditioned medium of TDSCs on tenocyte differentiation, migration, and transition to a fibroblastic phenotype in vitro. Successful isolation of exosomes from TDSCs was confirmed by high expression levels of CD81, CD63, CD9, and TSG101. Treatment with TDSC-derived exosomes promoted the growth and migration of cultured rat tenocytes, and increased the levels of the fibrosis markers collagen I, collagen III, scleraxis, tenascin C, and *α*-smooth muscle actin. Furthermore, vascular endothelial growth factor A (VEGFA) expression was higher in TDSC-derived exosomes than in TDSCs, and genetic knockdown of VEGFA suppressed the stimulatory effect of TDSC-derived exosomes on tenocyte development. Overall, these results demonstrate that VEGFA-enriched exosomes isolated from TDSCs promote differentiation and migration of cultured tenocytes and their transition to a fibroblastic phenotype. These data provide a new potential clinical treatment strategy for tendon injury.

## 1. Introduction

Rotator cuff tear (RCT) is one of the most common clinical injuries seen in orthopedic practice and sports medicine. The prevalence of RCT in various populations has been estimated to be approximately 20% [1, 2]. RCT is particularly common in elderly patients and can result in acute or chronic joint pain or other tissue injuries [3, 4]. In particular, RCT can cause substantial shoulder joint pain and dysfunction, and thereby impact an individual's quality of life and ability to work [5]. A variety of factors perturb RCT healing, including tendon degeneration, large tear size, and advanced age [6–8]. The incidence of RCT rerupture is relatively high because of the incomplete healing of tendon bone injury; therefore, it is of great importance to explore the mechanisms underlying tendon injury and identify new strategies for clinical treatment.

Tenocytes and immature tenoblasts are the major cell types in tendon tissue. Mature tenocytes are typically quiescent, nondividing cells that synthesize collagen, extracellular matrix molecules, and other components [9]. Degradation of these cells has been reported in rotator cuff-related diseases [10], and tenocyte proliferation, migration, and fibrosis greatly contribute to tendon repair [11, 12]. Novel treatment approaches for tendon injuries that aim to induce development of tenocytes into tenoligamentocytes have been reported [13].

Several donor cell types, including peripheral blood-derived mesenchymal stem cells (MSCs) [14], bone marrow-derived mesenchymal stem cells (BMSCs) [15, 16], dermal fibroblasts [17], and tenocytes [18], regulate tendon healing. Tendon-derived stem cells (TDSCs) can be isolated from tissues of humans and many other animals [19–21]. These precursor cells can differentiate into a variety of cell types, such as tenocytes, chondrocytes, osteocytes, and adipocytes [22]. Notably, TDSCs have a greater potential to generate tendon than other donor cells such as BMSCs [19, 21]. Application of donor cells directly to a lesion area has several limitations. For example, tenocytes produce a low level of collagen and exhibit poor differentiation [23], while BMSCs create ectopic bones and tumors [24].

Exosomes mediate cellular communication and molecular transport, and are crucial regulators of biological processes [25]. MSC-derived exosomes target the NLRP3 pathway to inhibit inflammatory responses in intervertebral disc degeneration [26] and have a potential application for tissue regeneration [27]. Thus, application of exosomes isolated from embryonic stem cells may be an effective method to treat tendon injury. However, there are few reports describing the targeting and regulation of tenocytes by TDSC-derived exosomes.

Vascular endothelial growth factor A (VEGFA), a member of the VEGF family of proteins, promotes angiogenesis, matrix formation, and collagen formation, all of which are important for tendon repair [28]. VEGFA in exosomes derived from stem cells is involved in a variety of bone functions and is reportedly upregulated in an animal model of osteoarthritis of the knee [29]. Notably, a recent study reported that VEGFA-enriched exosomes from cortical bone-derived MSCs stimulated by a CTRP9 polypeptide exert proangiogenic, antifibrotic, and cardioprotective effects [30]. However, whether VEGFA is enriched in TDSC-derived exosomes and its potential role in tenocyte function remain to be explored.

Here, we found that TDSC-derived exosomes are enriched with VEGFA and can regulate the migration, fibrotic activity, and proliferation of isolated rat tenocytes.

## 2. Materials and Methods

### 2.1. Ethics Statement and Animal Use

Sprague-Dawley (SD) rats were purchased from the Laboratory Animal Center of Jinan University, and the experiments were approved by the Ethics Committee of the First Affiliated Hospital, Jinan University. Rats were kept in a room with a light-controlled 12 h-12 h light-dark cycle, controlled room temperature (25°C), and unlimited food and water.

### 2.2. Isolation of Rat Tenocytes

Rotator cuff tendon tissues were isolated from SD rats as reported previously [31]. Tissues were sliced into small pieces, dispersed, and cultured in 6-well plates with Dulbecco's Modified Eagle Medium (DMEM, #11965092; Gibco, Waltham, MA, USA) supplemented with 10% fetal bovine serum (FBS, #10100147C, Gibco), 100 U/ml penicillin (#10378016, Gibco), and 100 U/ml streptomycin (#10378016, Gibco) in a humidified 5% CO_2_ incubator at 37°C for 5 days. Following trypsinization, tenocytes were placed in DMEM containing 10% FBS and passaged three times before use.

### 2.3. Isolation of TDSCs

TDSCs were harvested from Achilles tendon tissues of SD rats as reported previously [32]. Briefly, rat Achilles tendons were isolated and then incubated with collagenase (Sigma, Carlsbad, CA, USA) for 2 h at 37°C before harvesting TDSCs. Isolated cells were plated in 100 mm dishes at a density of 200 cells/cm^2^ and cultured in DMEM containing 20% FBS (Gibco), 100 U/ml penicillin, and 100 U/ml streptomycin (Gibco) in a standard tissue culture incubator for 10 days. Cells were passaged up to three times before use. TDSCs were identified as reported previously [32]. Expression of stem cell surface markers on TDSCs was measured by flow cytometry with antibodies against CD45 (ab40763; Abcam, Cambridge, UK), CD34 (ab81289, Abcam), CD90 (ab33694, Abcam), CD44 (12-0444-80; eBioscience, Thermo Fisher Scientific, MA, USA), and CD160 (ab274374, Abcam). The percentages of positive cells were measured with the FACScan system (Becton Dickinson, San Jose, CA, USA).

### 2.4. Isolation of TDSC-Derived Exosomes

To extract exosomes, after culture of TDSCs for 48 h, culture medium collected from 150 cm^2^ dishes was centrifuged at 300 × g for 20 min, 2000 × g for 10 min, and 10,000 × g for 60 min at 4°C. The supernatant was filtered with a 0.22 *μ*m filter (Merck-Millipore, MA, USA), ultracentrifuged at 100,000 × g for 1 h at 4°C, and resuspended in 200 *μ*l phosphate-buffered saline. The morphology of isolated exosomes was assessed by transmission electron microscopy (TEM), and their size was measured using NanoSight viewer (Malvern Instruments, Malvern, UK). The concentration of exosomes (i.e., the protein concentration in exosomes) was measured using a BCA Protein Kit (#P0009; Beyotime, Shanghai, China). Western blotting with primary antibodies against the exosome markers TSG101 (ab125011), CD81 (ab109201), CD63 (ab108950), and CD9 (#ab92726, all from Abcam) was performed. Extracted exosomes (20 *μ*g/ml) were added to the culture for treatment of tenocytes. The design of the procedures is shown in Figure 1(a).

### 2.5. Generation of Stable TDSCs

VEGFA-targeting shRNA sequences (shVEGFA) and a nonspecific shRNA (shNC) were subcloned into the lentiviral vector pLKO.1. HEK293 cells were transfected with the constructs for virus packaging. To remove cell debris from retrovirus-containing supernatants, 0.45 *μ*m Millex-HV filters (Millipore,) were used. TDSCs were infected with a lentivirus harboring shVEGFA, shNC, or vector control to generate stable cell lines. For selection, cells were treated with 2 *μ*g/ml puromycin (Sigma) for 48 h postinfection. The efficiency of VEGFA knockdown was determined by qPCR. The VEGFA shRNA sequences were 5′-GATCCGGCCAGCACATAGGAGTTCAAGAGAAGATTCAAGACGTCTCTCCTATGTGCTGGCCTTTTTTGTCGACA-3′ (sense) and 3′-GCCGGTCGTGTATCCTCAAGTTCTCTTCTAAGTTCTGCAGAGAGGATACACGACCGGAAAAAACAGCTGTTCGA-5′ (anti-sense) [33].

### 2.6. MTT Assay

Growth and proliferation of tenocytes were determined by an MTT assay. Briefly, tenocytes were seeded at a density of 1 × 10^4^/well into 96-well plates and cultured for the indicated duration. Subsequently, cells were treated with 50 *μ*l of 2 mg/ml MTT at 37°C for 2 h. After dissolving formazan crystals, absorbance at 570 and 620 nm was measured using a Chameleon™ multitechnology microplate reader (Hidex, Turku, Finland).

### 2.7. Transwell Assay

A transwell system (Corning, Lowell, MA, USA) was used to monitor the migration ability of tenocytes. Cells were suspended in RPMI medium after transfection and cultured in the upper chamber. The lower chamber contained medium with exosomes from TDSCs or control (normal culture medium). The upper chamber surface was cleaned with a cotton swab after incubation for 24 h. Under an optical microscope (IX81; Olympus, Tokyo, Japan), migrated cells were assessed following staining with 0.1% crystal violet for 10 min. Five randomly selected images per well were captured with a microscope, and migrated cells were counted in a blinded manner.

### 2.8. RNA Isolation and Real-Time qPCR

The expression levels of mRNAs encoding collagen I, tenascin C (TnC), collagen III, scleraxis (Scx), *α*-smooth muscle actin (*α*-SMA), and VEGFA were determined by real-time qPCR. Briefly, TRIzol reagent (Sigma) was applied to extract total RNA, reverse transcription was performed with EasyScript cDNA Synthesis SuperMix (TransGen Biotech, Beijing, China), and real-time qPCR was performed with TransStart Top Green qPCR SuperMix (TransGen Biotech). Relative expression levels were determined using the 2^-*ΔΔ*Ct^ method, and GAPDH was used as the control. The primer sequences are shown in Table 1.

### 2.9. Western Blotting

Proteins in samples lysed using ice-cold RIPA buffer (Beyotime) containing protease inhibitors (Invitrogen, Carlsbad, USA) were separated by 10% SDS-PAGE and transferred to PVDF membranes (Millipore). After blocking in milk for 40 min, membranes were incubated with primary antibodies against collagen I (#ab34710), Scx (#ab58655), *α*-SMA (#ab32575), TnC (#ab108930), collagen III (#ab7778), GAPDH (#ab8245), and VEGFA (#ab46154, all from Abcam). Following incubation with a secondary antibody (Abclonal Biotechnology, Cambridge, MA, USA), bands were detected by enhanced chemiluminescence (Beyotime).

### 2.10. Statistical Analyses

Each experiment was performed in triplicate. Data were analyzed with SPSS (27.0) to determine the mean and standard deviation. When comparing unpaired samples, the Student's t-test was used to compare two groups and a one-way analysis of variance was used to compare the means among three or more groups. *P* <0.05 was considered statistically significant.

## 3. Results

### 3.1. Generation and Identification of TDSC-Derived Exosomes

TDSCs were isolated from the Achilles tendons of SD rats and cultured. During culture, TDSCs displayed shuttle, spindle, and polygonal morphologies. Flow cytometry revealed that TDSCs highly expressed MSC markers, including CD90 (94.4%), CD44 (96.6%), and CD106 (97.3%) but not CD45 (0.3%) or CD34 (0.2%) (Figure 1(b)), as reported previously [34–36]. Exosomes were extracted from cultured TDSCs by ultracentrifugation. Their morphology and size were analyzed using TEM and NanoSight viewer, respectively. TEM showed that exosomes had a hollow spherical shape, and that their diameter was around 110 nm (Figure 1(c)). Western blotting showed that expression of the exosome markers CD9, CD81, CD63, and TSG101 was higher in the TDSC-derived exosome fraction than in the TDSC fraction (Figures 1(d) and 1 (e)). These data suggest that exosomes were successfully isolated from conditioned medium of TDSCs.

### 3.2. TDSC-Derived Exosomes Promote Tenocyte Differentiation, Migration, and Transition to a Fibroblastic Phenotype

An MTT assay revealed that treatment with TDSC-derived exosomes significantly promoted growth of tenocytes (Figure 2(a)). In addition, a transwell assay revealed that the migration ability of tenocytes treated with TDSC-derived exosomes was superior to that of untreated tenocytes (Figures 2(b)– 2(c)). The mRNA and protein levels of the fibrosis markers collagen I, collagen III, *α*-SMA, Scx, and TnC were determined in untreated and TDSC-derived exosome-treated tenocytes. The mRNA levels were significantly upregulated in tenocytes treated with TDSC-derived exosomes (Figures 2(d)). The protein levels showed the same trend as the mRNA levels (Figures 2(e) and 2(f), indicating that treatment with TDSC-derived exosomes promotes the transition of tenocytes to a fibroblastic phenotype. Taken together, these data suggest that TDSC-derived exosomes regulate the differentiation and migration of tenocytes and their transition to a fibroblastic phenotype.

### 3.3. VEGFA Is Upregulated in TDSC-Derived Exosomes and Tenocytes Treated with these Exosomes

To elucidate the mechanism underlying the growth-promoting effect of TDSC-derived exosomes on tenocytes, we performed qPCR analyses of various genes in TDSC-derived exosomes and tenocytes treated with these exosomes. The mRNA and protein levels of VEGFA were markedly higher in TDSC-derived exosomes than in the control group (Figures 3(a)– 3(c)). Furthermore, the mRNA and protein levels of VEGFA were markedly higher in tenocytes treated with TDSC-derived exosomes than in untreated tenocytes (Figures 3(d)– 3(f)). These results suggest that VEGFA is upregulated in TDSC-derived exosomes and tenocytes treated with these exosomes.

### 3.4. Genetic Knockdown of VEGFA Abolishes the Effects of TDSC-Derived Exosomes on Tenocyte Differentiation, Migration, and Transition to a Fibroblastic Phenotype

To confirm the effect of exosomal VEGFA on tenocytes, we constructed a TDSC line in which VEGFA was knocked down using a lentiviral shRNA (shVEGFA, Figure 4(a)). A TDSC line expressing a nonspecific shRNA (shNC) was generated as a control. Successful knockdown of VEGFA was confirmed by western blotting (Figure 4(b)). Exosomes were extracted from both these cell lines and added to tenocyte cultures. Exogenous VEGFA was added to tenocytes as a positive control. Treatment with VEGFA or exosomes derived from shNC-TDSCs significantly promoted the growth and migration of tenocytes (Figures 4(c)– 4(e)). However, knockdown of VEGFA abolished the stimulatory effect of TDSC-derived exosomes on growth (Figure 4(c)) and migration (Figures 4(d)–4(e)) of tenocytes. Furthermore, treatment of tenocytes with shNC-TDSC-derived exosomes or VEGFA significantly increased the levels of collagen I, *α*-SMA, collagen III, Scx, and TnC, whereas treatment with shVEGFA-TDSC-derived exosomes did not (Figures 4(g)– 4(h)). Overall, these results indicate that VEGFA promotes tenocyte growth, migration, and transition to a fibroblastic phenotype, and that the stimulatory effects of TDSC-derived exosomes on these behaviors of tenocytes are mediated via upregulation of VEGFA.

## 4. Discussion

Tenocytes play an important role in the repair of tendon injuries because they are the main cell type in tendon tissue. The results presented here demonstrate that TDSC-derived exosomes promote the growth and migration of rat tenocytes and their transition to a fibroblastic phenotype. VEGFA was upregulated in TDSC-derived exosomes and tenocytes treated with these exosomes, and silencing of VEGFA abolished the stimulatory effects of TDSC-derived exosomes on the behaviors of tenocytes. Taken together, these results suggest that VEGFA in TDSC-derived exosomes plays a novel role in regulating differentiation of tenocytes.

Exosomes isolated from various cell types can induce musculoskeletal tissue repair. For example, exosomes isolated from BMSCs promote myogenesis and muscle differentiation in a mouse injury model [37]. In addition, exosomes secreted during the transformation of myoblasts into myotubules promote myogenesis of adipose-derived stem cells and induce myofiber regeneration for injury repair [38]. Exosomes might also offer a novel way to treat osteoporosis. Exosomes derived from MSCs in a scaffold promote repair of bone defects via the PI3K/Akt pathway [39]. BMSC-derived exosomes improve osteoporosis by suppressing cell apoptosis and promoting osteoblast proliferation [40, 41]. In addition, a recent study found that exosomes secreted by endothelial cells improve osteoporosis by inhibiting osteoclast activity, and that this effect is superior to that of BMSC-derived exosomes [42]. Furthermore, exosomes are related to cartilage regeneration and osteoarthritis. Embryonic MSC-derived exosomes induce cartilage repair by increasing chondrocyte proliferation, enhancing collagen production, and regulating immune reactivity [43, 44]. miR-100-5p in exosomes derived from fat pad MSCs maintains cartilage homeostasis by regulating the autophagy pathway [45].

In view of their superior clonogenicity and tenogenic proliferation potential, TDSCs were selected as an ideal source of exosomes to manipulate the function of tenocytes in the current study. Exosomes isolated from TDSCs promote the tenogenesis of resident TDSCs, and regulate synthesis and degradation of the tendon matricellular matrix [46]. TDSC-derived exosomes suppress inflammation in a model of Achilles tendon injury [47]. Moreover, TDSC-derived exosomes promote growth and migration by modulating the transforming growth factor signaling pathway and promote tendon repair through miR-144-3p in TDSCs [35]. Here, we found that high expression of VEGFA is responsible for the stimulatory effects of TDSC-derived exosomes on tenocyte proliferation, migration, and transition to a fibroblastic phenotype because shRNA-mediated knockdown of VEGFA abolished the ability of TDSC-derived exosomes to promote tenocyte development. VEGF is critical for bone tissue repair. Expression of VEGF is upregulated in injured leg bones of rats and cruciate ligaments of dogs [48]. In addition, during acute injury healing, BEGF and VEGF are upregulated at the bone-tendon junction [28]. Recently, high expression of VEGF in MSCs was reported to regulate repair of RCT via regulation of miR-205-5p [49]. In addition, induction of VEGFA expression by engineered nanoparticles promotes tendon healing. In our previous study, we showed that the long noncoding RNA H19 accelerates differentiation of rat tenocytes by inhibiting miR-140-5p, which leads to upregulation of VEGFA at the lesion site [31]. Expanding on this finding, we demonstrated here that upregulation of VEGFA in exosomes from TDSCs promotes tenocyte development. Taken together, these findings suggest that VEGFA plays a critical role in tendon differentiation and repair. However, the detailed mechanism by which VEGFA is upregulated in TDSC-derived exosomes and the role of these exosomes in RCT repair require further investigation.

In summary, we demonstrated that VEGFA-enriched exosomes isolated from TDSCs promote growth and migration of rat tenocytes and their transition to a fibroblastic phenotype. Further studies of TDSC-derived VEGFA-expressing exosomes may provide new insights into novel approaches for the clinical treatment of tendon injury.

## Figures and Tables

**Figure 1:** Morphology and phenotypic identification of TDSCs and TDSC-derived exosomes. (a) Schematic presentation of the experimental design. (b) Flow cytometric analysis of cell surface markers of TDSCs. Red curves represent controls, and green curves represent surface markers. (c) TEM showing the morphology and size distribution of exosomes derived from TDSCs. Scale bar: 100 nm. (d) Western blot analyses of CD9, CD63, CD81, and TSD101 in exosomes isolated from cultured TDSCs. (e) Quantification of the expression levels of the proteins shown in (D). ∗*P* <0.05 relative to TDSCs.

**Figure 2:** TDSC-derived exosomes promote tenocyte differentiation, migration, and transition to a fibroblastic phenotype. (a) An MTT assay to investigate the proliferation of tenocytes in the control (normal culture medium) and TDSC-derived exosome-treated groups. (b) A transwell assay to monitor the migration of tenocytes in the control and TDSC-derived exosome-treated groups. (c) Quantification of the transwell assay data shown in (B). The mRNA (d) and protein (E-F) levels of collagen I, collagen III, *α*-SMA, Scx, and TnC in control and TDSC-derived exosome-treated tenocytes determined by RT-qPCR and western blotting. ∗*P* <0.05 relative to the control group.

**Figure 3:** VEGFA is upregulated in TDSC-derived exosomes and tenocytes treated with these exosomes. (A–C) The mRNA (A) and protein (B, C) levels of VEGFA in TDSCs and TDSC-derived exosomes determined by real-time qPCR and western blotting. (D–F) The mRNA (D) and protein (E, F) levels of VEGFA in control and TDSC-derived exosome-treated tenocytes determined by RT-qPCR and western blotting. ∗*P* <0.05, ∗∗*P* <0.01 relative to TDSCs or the control tenocyte group.

**Figure 4:** Genetic knockdown of VEGFA suppresses the stimulatory effects of TDSC-derived exosomes on tenocyte growth, migration, and transition to a fibroblastic phenotype. (A) TDSCs with VEGFA knockdown induced by a lentivirus and control TDSCs. (B) Knockdown of VEGFA determined by western blotting and quantification. Tenocytes were treated with VEGFA or exosomes derived from shVEGFA-TDSCs or shNC-TDSCs. (C) An MTT assay to investigate the growth of tenocytes. (D, E) A transwell assay to monitor the migration of tenocytes. (F–H) The mRNA (F) and protein (G, H) levels of collagen I, *α*-SMA, collagen III, Scx, and TnC determined by RT-qPCR and western blotting. ∗*P* <0.05, ∗∗*P* <0.01 relative to the indicated group.

**Table 1:** Real-time qPCR primer sequences (5'-3').

Gene	Forward primer	Reverse primer
*Vegfa*	GCACATAGGAGAGATGAGCTTCC	CACGCCTTGGCTTGTCACAT
*Scx*	AGCCCAAACAGATCTGCACCTT	CTTCCACCTTCACTAGTGGCATCA
*Collagen I*	GTCCGAGGTCCTAATGGAGATGC	GGTCCAGGGAATCCGATGT
*Collagen III*	ACAGCAGTCCAATGTAGATG	GAGCAGGTGTAGAAGGCTG
*α-SMA*	GAGGCACCACTGAACCCTAA	CATCTCCAGAGTCCAGCACA
*Tnc*	CGGGGCTATAGAACACCAGT	AACATTTAAGTTTCCAATTTCAGGTT
*Gapdh*	TGATTCTACCCACGGCAAGTT	TGATGGGTTTCCCATTGATGA

## Data Availability

The datasets used and/or analyzed during the current study are available from the corresponding author on reasonable request.
